The article "Concurrent malignant melanoma and cutaneous involvement by classical hodgkin lymphoma (CHL) in a 63 year-old man" was published in 2013. Journal: Diagn Pathol.

# Concurrent malignant melanoma and cutaneous involvement by classical hodgkin lymphoma (CHL) in a 63 year-old man

**DOI:** 10.1186/1746-1596-8-135

**Published:** 2013-08-09

**Authors:** Alejandro A Gru, Dongsi Lu

**Affiliations:** 1 Department of Pathology & Immunology, Washington University, St. Louis School of Medicine, St. Louis, MO, USA; 2 Department of Pathology, St. Luke Hospital, Chesterfield, MO, USA

**Keywords:** Malignant melanoma, Classical Hodgkin lymphoma, Bone marrow transplant

## Abstract

**Abstract:**

Classical Hodgkin lymphoma (CHL) is a lymphoproliferative disorder that has a bimodal age distribution, affecting young and elderly individuals, and is curable in more than 90% of patients. Here we report the coexistence of cutaneous CHL and malignant melanoma as the presentation of papules and a plaque, in an individual with remote history of systemic CHL. One of the biopsies showed a mononuclear cell infiltrate with Reed-Sternberg (RS) like cells that were positive for CD30 and CD15, but negative for CD45. A second concurrent biopsy showed an atypical melanocytic proliferation with significant pagetoid spreading and diffuse Melan-A staining. Based on morphology alone, it is almost impossible to distinguish CHL from other primary cutaneous lymphoproliferative disorders, such as CD30+ lymphoproliferative disorder (lymphomatoid papulosis (LyP) and primary cutaneous anaplastic large-cell lymphoma), or even tumor stage mycosis fungoides when the epidermotropism is minimal. Additionally, bizarre melanocytic cells can also appear similar to RS cells. Our case illustrates the first case report of malignant melanoma and CHL in a patient presenting simultaneously.

**Virtual slides:**

The virtual slide(s) for this article can be found here: http://www.diagnosticpathology.diagnomx.eu/vs/8979757349937225

## Introduction

Classical Hodgkin lymphoma (CHL) is a lymphoproliferative disorder that has a bimodal age distribution, affecting young and elderly individuals, and is curable in more than 90% of patients. It has a propensity to follow dissemination in a well-established pattern. This facilitates the use of localized treatment modalities in its therapeutic approach that include surgery and radiotherapy. Advanced stage presentations occur in less than 30% of patients, and the skin is only rarely affected. Isolated case reports of CHL affecting the skin have been described. However, CHL can have other cutaneous manifestations that may not be directly attributed to the dissemination of the disease. Here we report the coexistence of CHL and malignant melanoma as the presentation of papules and a plaque, in an individual with remote history of CHL. This is the first report of the simultaneous existence of both disorders.

The article "Concurrent malignant melanoma and cutaneous involvement by classical hodgkin lymphoma (CHL) in a 63 year-old man" was published in 2013. Journal: Diagn Pathol.

## Case presentation

A 62 year-old man presented with 3–4 months history of two pink-papules on the scalp, and a pink crusted plaque on the left neck. He had a previous remote history of nodular sclerosis classical Hodgkin lymphoma and therapy related acute myeloid leukemia with monosomy 7. His lymphoma was under control after the chemotherapy, but he did had bone marrow extension at the time of diagnosis. A hematopoietic allogeneic transplant was done after his original diagnosis of acute myeloid leukemia. Two punch biopsies were obtained. The biopsy from the left neck (Figure 1) showed a mixed dermal inflammatory infiltrate with scattered atypical large multinucleated and mononuclear cells, intermixed with aggregates of neutrophils, small lymphocytes and histiocytes. The mononuclear cells had hyperchromatic nuclei with vesicular smudged chromatin and prominent cherry red nucleoli, resembling Reed-Sternberg cells. By immunohistochemistry (Figure 2), the atypical cells were positive for CD30, CD20, CD79a, and had dim CD15 and PAX5 staining. They were negative for CD45. A CD3 and CD43 highlighted the abundant intermixed T-cells, but were negative among the atypical large cells. CD68 stained a rich histiocytic background. A Melan-A and S100 stains were also negative. In-situ hybridization for EBV was negative as well.

**Figure 1:** **Punch biopsy from the left neck with involvement by HL.** 1**a** and 1**b**: Hemotoxylin and Eosin stain (20× and 100×). There is an atypical infiltrate involving the entire dermis with scattered larger cells. A grenz-zone is between the infiltrate and the epidermis. 1**c** – 1**f**: Hemotoxylin and Eosin stain (200× and 400×). The infiltrate is composed predominantly of small lymphocytes and abundant histiocytes in the background. Several large cells, some of which are binucleated and show prominent nucleoli (compatible with Reed-Sternberg cells and RS variants) are seen. In addition, scattered neutrophils are also present. Atypical mitoses can be easily detected.

**Figure 2:** **Immunohistochemistry of the punch biopsy from the left neck.** The atypical cells are positive for CD30, CD79a and CD20. CD15 and PAX5 show positive and dim staining in the tumor cells. CD3 and CD68 (not shown) stain a background of small T-cells and abundant histiocytes, respectively. The large cells are negative for CD45, EBER and Melan-A (not shown).

The two biopsies from the scalp (Figure 3) show an atypical melanocytic proliferation, with features most compatible with malignant melanoma, largely involving the dermis. There were large nests of atypical melanocytes with light eosinophilic cytoplasm, hyperchromatic and vesicular nuclei with variable prominent nucleoli. Scattered mitotic figures were seen, including in the deeper portion of the lesion. No maturation towards the base of the lesion was seen. An intraepidermal melanocytic component was present in one of the biopsies. No perineural or lymphovascular space invasion was identified. Immunohistochemistry for Melan-A and HMB-45 confirmed the melanocytic origin of the tumor cells.

The article "Concurrent malignant melanoma and cutaneous involvement by classical hodgkin lymphoma (CHL) in a 63 year-old man" was published in 2013. Journal: Diagn Pathol.

**Figure 3:** **Punch biopsy from the scalp with malignant melanoma.** 3**a** and 3**b**: Hemotoxylin and Eosin stain (20× and 100×). There is an atypical melanocytic proliferation with a predominant dermal component, but with individual atypical junctional nests seen. 3**c** and 3**d**: Hemotoxylin and Eosin stain (200× and 400×). The atypical melanocytes are predominantly epithelioid with light eosinophilic cytoplasm, hyperchromatic and vesicular nuclei with variable prominent nucleoli. Scattered mitotic figures were seen, including in the deeper portion of the lesion. 3**e** and 3**f**: Melan-A immunostain (20× and 100×).

## Discussion

Hodgkin lymphoma (HL) is a disease of young adults (12% of all lymphomas) and elderly people, and is composed of two separate entities: classical HL (95% of cases) and nodular lymphocytic predominant HL (5% of cases) [1]. First described by the German physician Grosz in 1906, cutaneous Hodgkin lymphoma (CHL), an exceedingly rare manifestation of the disease (0.5 – 7.5 %), occurs when the malignant cells invade the dermis [2]. Nonetheless, cutaneous symptoms can be seen in up to 40% of patients with HL [3]. The current WHO-EORTC classification identifies cutaneous HL as a secondary systemic dissemination of the disease [1,4]. Cutaneous manifestation of HL show different clinical features: (a) papules, (b) plaques, (c) nodules or tumors, (d) ulcerative lesions, (e) various combinations of these features and (f) erythroderma [2]. It is usually centered in the reticular dermis and commonly extends into the subcutaneous fat. The tumor shows nodular or interstitial growth pattern with adnexal involvement. Various forms of Reed- Sternberg cells with large, hyperchromatic, irregular shaped nuclei are easily identifiable. The Reed-Sternberg cells are admixed predominantly with plasma cells and lymphocytes with occasional histiocytes and eosinophils. Necrosis is generally absent. The epidermis is spared in most of the cases [2-5]. In this particular case, the patient had a remote history of nodular sclerosis classical Hodgkin lymphoma that preceded the secondary involvement of the skin by many years (10–15 years). Although his original biopsy slides were not available for review, the histologic features seen on the diagnostic skin biopsy were more suggestive of a mixed cellularity variant of CHL: there was an abundance of mixed inflammatory cells that included neutrophils, histiocytes, plasma cells, lymphocytes, and rare eosinophils without significant fibrosis. The population of RS cells and variants was significant as it is depicted on the Figure 1.

The article "Concurrent malignant melanoma and cutaneous involvement by classical hodgkin lymphoma (CHL) in a 63 year-old man" was published in 2013. Journal: Diagn Pathol.

Based on morphology alone, it is almost impossible to distinguish CHL with abundant numbers of neoplastic cells from other primary cutaneous lymphoproliferative disorders, such as CD30+ lymphoproliferative disorder (lymphomatoid papulosis (LyP) and primary cutaneous anaplastic large-cell lymphoma (ALCL)), or even tumor stage mycosis fungoides when the epidermotropism is minimal. Other reactive CD30+ processes including: pseudolymphomatous drug reactions, nodular scabies, atopic dermatitis, and infections can also be in the differential diagnosis [4].

By immunohistochemistry, the neoplastic cells in Classical HL are positive for CD30 in nearly all cases and CD15 for the majority (75–85%) of cases and are usually negative for CD45, CD20, ALK and EMA. However, up to 20-30% of CHL can be positive for CD20, and its positivity is a marker of better prognosis, and response to rituximab. The B-cell nature of Reed-Sternberg cells is shown by the B-cell specific activator protein (BSAP), product of the PAX-5 gene in approximately 90% of cases. Additionally the tumor cells can be positive for EBER, by in-situ hybridization [1,5,6]. Other immunohistochemical markers that have some utility are OCT-2 and BOB-1, which are positive (not both) in up to 90% of cases [1]. In contrast, LyP, c-ALCL, or transformed MF show invariable negative expression of CD15 or Pax-5 [4,6]. A systemic B-cell lymphoma that can sometimes enter in the differential diagnosis is T-cell histiocyte-rich large B-cell lymphoma (THRLBCL). But in THCRLBCL there is strong expression of CD45, CD20, CD79a and PAX-5. The current case showed a typical CHL immunophenotype with CD30 and CD15 expression, but negative for CD45. An unusual phenotype with CD20 and CD79a expression was also seen, but PAX5 showed the classic dim staining characteristic of CHL. EBER was negative, a feature commonly seen in most cases of nodular sclerosis and mixed cellularity CHL.

The mode of HL spread to the skin has been explained by three mechanisms: (1)retrograde lymphatic spread, distal to the tumor involved regional lymph node(s), which is the most common; (2)direct extension from an underlying nodal focus; and (3) hematogenous dissemination where no tumor-involved lymph nodes are identified in the immediate vicinity of the involved skin [3,4].

The article "Concurrent malignant melanoma and cutaneous involvement by classical hodgkin lymphoma (CHL) in a 63 year-old man" was published in 2013. Journal: Diagn Pathol.

The coexistence of different malignancies in patients with Hodgkin and NHL has been previously documented: Yang et al. [7] reported a patient with nodal angioimmunoblastic T-cell lymphoma (AITCL) who had a partial response to chemotherapy, and developed an EBV-associated cutaneous diffuse large B-cell lymphoma few months after his original diagnosis of AITCL. El Demellawy et al. [8] reported a synchronous collision tumor of malignant melanoma and chronic lymphocytic leukemia/small lymphocytic lymphoma (CLL/SLL). We have also seen in our personal experience the coexistence of CLL/SLL with melanoma and squamous cell carcinoma.

Concurrent malignant melanoma and lymphoma occurs in 0.3% of patients with melanoma [9]. Since 1960, a rising incidence of melanoma and NHL has been observed, probably related to UV exposure and immunosupression (such as cases presenting in individuals who are stem cell transplant recipients and patients with AIDS) [9,10]. Adami et al. [10] first reported a link between NHL, CLL/SLL and skin cancer (the relative risk of developing melanoma was 2.4 among NHL patients) and suggested that UV light may contribute to increasing incidence of NHL. Riou et al. [11] reported a 16 fold higher incidence of lymphomas in patients with malignant melanoma. A recent study also found a 3.5 to 7.5 fold increase of NHL in patients with melanoma [9]. Alterations of p16 pathway, which inhibit CDNK4, a tumor suppressor gene, are common in both types of malignancies [5,9].

More interestingly, the development of skin cancers after non-myeloablative allogeneic bone marrow transplants (NMAT) has been well documented. Cavalier et al. [12] reported a series of 6 cases of skin cancers (mostly squamous cell carcinomas, but 2 of the patients had melanoma) in patients with NMAT. The most interesting finding in their study was a particular strong association of skin cancers in those patients who received their transplant for myelodysplasia or acute myeloid leukemia. In this case the patient developed a therepy related myeloid neoplasm subsequent to the chemotherapy for CHL. The mechanism implicated in the development of skin cancers is the immunosupression from the induction chemotherapeutic regimens that are administered prior to the transplant. In particular, the depletion of CD4+ lymphocytes is a well known predisposer for skin cancers. Patients who have an aggressive myeloid neoplasm usually receive more intensive induction regimens, a fact that creates a more immunosuppressive background. Ultimately, fludarabine, a purine analogue that is typically use in induction chemotherapy, results in DNA inactivation and apoptosis. Fludarabine also inhibits DNA-polymerase, RNA-polymerase, DNA-ligase, DNA-primase and ribonucleotide reductase [13]. Fludarabine also depletes CD3, CD4 and CD8 lymphocytes over a period of a month. In this case fludarabine was one of the drugs administered prior to his transplant. Additional possible mechanisms which are linked to carcinogenesis include p53 mutations and HPV infection (in squamous cell carcinomas).

The article "Concurrent malignant melanoma and cutaneous involvement by classical hodgkin lymphoma (CHL) in a 63 year-old man" was published in 2013. Journal: Diagn Pathol.

In the past, 3 cases of patients with melanoma developed Hodgkin’s disease thereafter and were published in the literature [7,9]. However, concurrent cutaneous involvement by HL and melanoma has never been reported. Causality between both malignancies remains to be established. Our case illustrates the first case report of malignant melanoma and CHL in a patient presenting simultaneously.

### Consent

An attempt to obtain informed consent was performed. However, this patient has been lost to follow up, and no close family members were available (based on the provided demographic information) to obtain informed consent from.

## Competing interests

The authors don’t have any conflict of interest to disclose.

## Authors’ contributions

AAG wrote the manuscript, took the clinical pictures, obtain the references, was responsible for the additional work-up performed after the manuscript acceptance, and also edited it. DL was the main pathologist who had the case and review the manuscript and performed additional editing. All authors read and approved the final manuscript.
